The article "Time-Frequency Analysis of EEG Signals and GLCM Features for Depth of Anesthesia Monitoring" was published in 2021. Journal: Comput Intell Neurosci.

# Time-Frequency Analysis of EEG Signals and GLCM Features for Depth of Anesthesia Monitoring

**DOI:** 10.1155/2021/8430565

**Published:** 2021-08-11

**Authors:** Seyed Mortaza Mousavi, Akbar Asgharzadeh-Bonab, Ramin Ranjbarzadeh

**Affiliations:** ^1^Department of Biomedical Engineering, Urmia Medical Sciences University, Urmia, Iran; ^2^Department of Electrical and Computer Engineering, Urmia University, Urmia, Iran; ^3^Department of Telecommunications Engineering, Faculty of Engineering, University of Guilan, Rasht, Iran

## Abstract

One of the important tasks in the operating room is monitoring the depth of anesthesia (DoA) during surgery, and noninvasive techniques are very popular. Hence, we propose a new scheme for DoA monitoring considering the time-frequency analysis of electroencephalography (EEG) signals and GLCM features extracted from them. To this end, at first, the time-frequency map (TFM) of each channel of each EEG is computed by smoothed pseudo-Wigner–Ville distribution (SPWVD), where the EEG signal used in this paper is recorded in 15 channels. After that, we consider the gray-level co-occurrence matrix (GLCM) to obtain the content of TFM, and after that, four features such as homogeneity, correlation, energy, and contrast are obtained for each GLCM. Finally, after the selection of efficient features using the minimum redundancy maximum relevance (MRMR) method, the K-nearest neighbor (KNN) classifier is utilized to determine the DoA. Here, we consider the three states, namely, deep hypnotic, surgical anesthesia, and sedation and awake states according to bispectral index (BIS), and each EEG epoch is classified to these states. We also employ data augmentation to enhance the training phase and increase accuracy. We obtain the accuracy and confusion matrix of the proposed method. We also analyze the effects of a number of gray levels of GLCM, distance measure in KNN classifier, and parameters of data augmentation on the performance of the proposed method. Results indicate the efficiency of the proposed method to determine the DoA during surgery.

## 1. Introduction

General anesthesia (GA) is a necessary state for many surgical procedures. There are several essential features of anesthesia which are displayed by patients. Some of these features are the lack of movement, awareness, and recall of the surgical intervention as well as unresponsiveness to painful stimuli [1, 2]. As overly light anesthesia is the most common cause of awareness, anesthesiologists use several indicators to measure the depth of anesthesia (DoA). A continuum of progressive central nervous system (CNS) depression and decreased responsiveness to stimulation is referred to as DoA or depth of hypnosis [3, 4].

One of the most forlorn and fearsome senses is awareness during anesthesia. It is a complication with potential long-term psychological consequences like posttraumatic irritability, stress, and anxiety [5]. Monitoring DoA is a solution to this issue. The most important task in the operational room is preventing excessive DoA or awareness and improving patients' outcomes which can be performed by precise drug delivery to the patients. An accurate evaluation of DoA can help us to this end [6].

Numerous approaches and devices were designed and produced to assess DoA. These devices work based on clinical/conventional monitoring and/or brain electrical activity monitoring, and each of them has its special drawbacks. Previous studies demonstrate that since CNS is the final target for GA drugs, the electroencephalogram (EEG) signal can be more informative for the determination of DoA compared to those works just based on simple vital signs. BIS [7], auditory evoked potential (AEP) monitors [8], entropy [9], and narcotrend [10] are some of EEG-based commercially DoA monitors. It turned out that these devices are not exactly accurate and suffer from several drawbacks.

Recently, several works aimed at introducing new methods to measure the DoA. Bayesian techniques were employed in [11] to the assessment of DoA, where the limiting large-sample normal distribution was considered, and it was shown that the maximum a posteriori (MAP) values increase gradually as the anesthesia states change from awake to light, moderate, and deep anesthesia. Distinguishing awake states from GA using EEG signals was the aim of authors in [12]. They extracted 11 features from EEG signals such as entropy, fractal, and spectral, and then, efficient ones were selected. It was found that entropies including permutation and sample, Beta-index, and detrended fluctuation analysis yield the highest accuracy with a classifier based on the adaptive neuro-fuzzy inference with linguistic hedges. Quasi-periodicities in EEG were used for analyzing the variations of DoA in [13]. To this end, phase-rectified signal averaging was employed. The results indicated that this method achieves better results than the sample and permutation entropies.

The six features including beta ratio, spectral edge frequency, and four bands of spectral energy were extracted from the EEG signal, and then, the decision tree classifier was used to determine the DoA in [14]. The authors considered the four classes for DoA as deep, moderate, and light versus awake state. In [15], at first, the noise removal from EEG signals was performed by Hurst's method, and the maximum of Hurst's ranges was considered as EEG response. Then, it was shown that maximum PSD can be used to distinct transitions of DoA states. Atomic decomposition was considered in [16] to decompose the EEG signals. Then, several features were extracted from decomposed subbands, and the SVM classifier discriminates between awake and sedated states.

The near-infrared spectroscopy (NIRS) signals were considered for recording the cerebral hemodynamic variables in [17] to monitor the DoA. The authors proposed to measure the sample entropy to describe the complexity information of cerebral hemodynamic variables. The multimodal system, which simultaneously uses the EEG and NIRS signals, was considered in [18] to monitor the DoA. It was shown that, with the EEG + NIRS signals, the clinically important transition from the awake to deep state can be detected, while transition in a clinical trial cannot be detected by BIS.

Ordinal power spectral density (O-PSD) was introduced in [19] for measuring the DoA. A deep neural network (DNN) named AnesNet was introduced in [20] to quantify the DoA. The raw EEG signals were given to a convolutional neural network (CNN) with convolution, pooling, and fully connected layers to determine the DoA. In [21], short-time Fourier transform (STFT) was employed for obtaining PSD, and CNN determines the DoA according to the given PSD. The wavelet transform was employed in [22] for analyzing the DoA from EEG signals. For this purpose, extracted features were clustered using a classifier based on the wavelet. Also, the specifications of eigenvectors were considered for extracting the specs of the midlatency auditory evoked EEG under anesthesia.

Since EEG signals present nonlinear characteristics in anesthesia conditions [23], we present a method for DoA monitoring considering the time-frequency analysis of EEG signals. We employ the smoothed pseudo-Wigner–Ville distribution (SPWVD) [24] to obtain a time-frequency map (TFM) of EEG epochs. In order to obtain the characteristics of TFM, we employ the gray-level co-occurrence matrix (GLCM) and, then, extract four features from it. Since all extracted features are not informative, we employ minimum redundancy maximum relevance (MRMR) to select the efficient ones from the feature vector. Finally, the K-nearest neighbor classifier (KNN) determines the depth of anesthesia. We also utilize the data augmentation by adding zero-mean white Gaussian noise to training samples in order to enhance the generality of the trained classifier. Hence, the contributions of this research can be summarized as follows:

- Employing SPWVD for obtaining the TFM of EEG signals
- Employing GLCM features in order to describe the time-frequency content
- Feature selection by MRMR algorithm to reduce the complexity of classification
- Employing data augmentation to increase the generality of KNN classifier
- Obtaining the accuracy and confusion matrix of the proposed scheme
- Analyzing the accuracy for different distance measures as well as different number of gray levels and augmentation parameters

Following this introduction, Section 2 describes the recorded EEG signals which are used in this research.  Section 3 explains the proposed for monitoring DoA in detail.  Section 4 contains the results and eventually.  Section 5 presents the concluding remarks and the directions of future works.

## 2. Data

Six female participants aging in the range 26–72 years old, with a mean of 45.5 years old, were contributed in order to record the required data. These participants were scheduled for elective gynecological surgeries. It should be mentioned that this research was approved by the Institutional Research Ethics Committee. According to the American Association of Anesthesiology physical status classification, all patients were in ASA I and ASA II. All patients confirmed informed consent before initiation of data recording [6].

In order to avoid unnecessary delays in the surgical program, the preoperation (Pre-Op) period started about an hour before surgery, and then, spontaneous EEGs were recorded for 5 minutes. After that, the patients were transferred to the operation room and electrodes of the BIS device were attached before starting the operational (OP) period. Spontaneous EEG signals were recorded during maintenance and emergence periods of anesthesia. A long recording was made ten minutes before the anesthesia was stopped and waking up.  Table 1 contains the duration of spontaneous EEG and BIS data recording during surgery for different patients [6].

The EEG electrodes were montaged according to the 10/20 standard to include 15 channels, namely, Fp1, Fp2, F7, F3, Fz, F4, F8, T7, C3, Cz, C4, T8, P3, Pz, and P4 [6]. Simultaneously, BIS was recorded in a parallel manner using the available anesthesia monitor (Aspect Medical Systems) and was considered as a reference. BIS index is in the range [0, 100], where 0 denotes full cortical silence and 100 is the fully awake state. The appropriate state for adequate surgical anesthesia is the BIS level between 40 and 60 [2].

The EEG signals were segmented into the epochs of 30 seconds, which have 50% overlap with each other. The average of BIS during each epoch was computed, and each was labeled as deep hypnotic (*D*), surgical anesthesia (*A*), and sedation and awake (*S*) considering the average BIS of an epoch. The epochs with the average BIS smaller than the 40 are labeled as D. The average BIS between 40 and 60 labels the epoch as A. The epochs with average BIS greater than 60 are called S. In Table 2, the numbers of epochs from each label for different subjects are reported.

## 3. Proposed DoA Monitoring

Figure 1 presents the procedure of the proposed scheme for DoA classification. As shown, the proposed scheme generally determines the DoA in three steps including preprocessing, feature extraction and selection, and classification, which are explained in detail in the following.

### 3.1. Preprocessing

At first, artifacts and corrupted BIS data were identified and removed manually from raw recorded signals. The frequency content of the cleaned data is in the range [0, 300] Hz and has a maximum amplitude of about 100 *μ*V. At first, a high-pass filter with a cutoff frequency of 0.5 Hz was employed to remove the disturbances at very low frequencies. Also, to remove the high-frequency noise, a low-pass filter with a cutoff frequency of 70 Hz was used. Furthermore, a notch filter with a null frequency of 50 Hz was employed to remove power supply noise. Since the maximum informative frequencies of EEG signals are less than 60 Hz, we consider the decimation to reduce the sampling frequency from 1000 Hz to 100 Hz, which reduces the computational complexity [21]. One epoch from states of overdeep, surgical anesthesia, and sedation and awake in different channels is shown in Figures 2–4 , respectively.

### 3.2. Feature Extraction

The proposed feature extraction in this paper employs the three steps as follows:

- Time-frequency analysis
- GLCM features
- Feature selection

In the following, we present each step in more detail.

#### 3.2.1. Time-Frequency Analysis

It was mentioned that EEG signals are not stationary and should be analyzed as pseudostationary signals. Therefore, traditional frequency-domain analysis tools such as Fourier transform cannot help to characterize it in the frequency domain. Hence, we should consider time-frequency transforms in order to obtain the frequency-domain content.

The first step for computing the WVD of a signal *x*(*t*) is obtaining its analytical signal as

(1) $$\begin{array}{c} y\left(t\right)=x\left(t\right)+j\hat{x}\left(t\right), \end{array}$$

where the Hilbert transform of *x*(*t*), i.e., $\hat{x}\left(t\right)$, is defined as

(2) $$\begin{array}{c} \hat{x}\left(t\right)=H\left[x\left(t\right)\right]=\frac{1}{\pi }\int_{-\infty }^{\infty }x\left(t\right)\frac{1}{t-\tau }\text{d}\tau . \end{array}$$

Accordingly, the Winger distribution is defined as

(3) $$\begin{array}{c} W_{x}\left(t,f\right)=\int_{-\infty }^{\infty }y^{*}\left(t-\frac{\tau }{2}\right)y\left(t+\frac{\tau }{2}\right)e^{-j2\pi f\tau }\text{d}\tau , \end{array}$$

where (·)^*∗*^ denotes the conjugate operation and $j=\sqrt{-1}$.

The Wigner–Ville distribution provides the energy density in the time-frequency domain. This distribution is one of the Cohen class distributions. Distribution smoothing should be applied to diminish the cross-term, which is the zero-density energy components of Winger distribution. Reducing the cross-term enhances the accuracy of distribution. In order to improve WVD, a smoothing function, either frequency or time smoothing function, can be added [25, 26].

Considering the frequency smoothing function *h*(*τ*), the pseudo-WVD (PWVD) is defined as

(4) $$\begin{array}{c} \text{PWVD}\left(t,f\right)=\int_{-\infty }^{\infty }h\left(\tau \right)y\left(t+\frac{\tau }{2}\right)y^{*}\left(t-\frac{\tau }{2}\right)e^{-j2\pi f\tau }\text{d}\tau . \end{array}$$

As the smoothing function *g*(*t*) is added in the time domain, the smoothed PWVD (SPWVD) is obtained as

(5) $$\begin{array}{c} \text{SPWVD}\left(t,f\right)=\int_{-\infty }^{\infty }h\left(\tau \right)\left(\int_{-\infty }^{\infty }g\left(t\right)y\left(t+\frac{\tau }{2}\right)y^{*}\left(t+\frac{\tau }{2}\right)\text{d}t\right)e^{-j2\pi f\tau }\text{d}\tau . \end{array}$$

It should be mentioned that both *h*(*τ*) and *g*(*t*) are rectangular windows.

EEG signals are recorded in 15 channels; hence, SPWVD should be calculated for each channel separately. The SPWVDs for different channels of one epoch from each class of subject 1 are shown in Figures 5–7 for deep hypnotic (*D*), surgical anesthesia (*A*), and sedation and awake (*S*) classes, respectively. The results show that the values of SPWVD are negligible for frequencies higher than 8 Hz. In other words, EEG signals have meaningful content in the delta and theta bands. Therefore, the SPWVD is given for the frequency range [0 8] Hz for better representation of EEG variations in the time-frequency plane. It is observed that the deep hypnotic epoch demonstrates the minimum activity compared to the surgical anesthesia and sedation and awake epochs. Because in this case person has the lowest activity and as observed EEG rhythms with frequencies lower than two Hz are dominant. Comparing Figure 6 with Figures 5 and 7 depicts that the EEG epoch from the surgical anesthesia class has higher activity in the frequency range in the band [0 8] Hz compared to surgical anesthesia and sedation and awake states. The activity in higher frequencies reduces in sedation and awake compared to the surgical anesthesia state, but it is higher than the deep hypnotic state.

(7) $$\begin{array}{c} E_{k}=\sum_{i=1}^{L}\sum_{i=1}^{L}G_{k}^{2}\left(i,j\right),\\ h_{k}=\sum_{i=1}^{L}\sum_{i=1}^{L}\frac{G_{k}\left(i,j\right)}{1+\left|i-j\right|}, \end{array}$$

#### 3.2.2. GLCM Features

As shown, the EEG epochs have different time-frequency contents during different levels of GA. Hence, we can use texture analysis methods to describe the time-frequency content. Several texture-based methods were introduced to obtain the content of images such as local binary pattern (LBP) [27–30], autocorrelation function (ACF) [31], binary Gabor pattern (BGP) [32], gray-level co-occurrence matrix (GLCM) [28, 33], and local spiking pattern (LSP) [34].

Different combinations of gray levels within the image can be described by GLCM which can be useful in the identification of the different regions of interest in the images. GLCM extracts the texture features considering the second-order relationship between reference and neighboring pixels [35, 36]. GLCM develops the co-occurrence matrix by comparing the pixel values of neighboring pixels, where the number of rows and columns of the matrix is equal to a number of gray levels. After computing GLCM for *k* th channel of EEG signal, i.e., **G**_*k*_, with *L* levels, four features are extracted from it including contrast (*c*_*k*_), correlation (*r*_*k*_), energy (*e*_*k*_), and homogeneity (*h*_*k*_) which are computed as follows [37]:

(6) $$\begin{array}{c} c_{k}=\sum_{i=1}^{L}\sum_{i=1}^{L}{\left(i-j\right)}^{2}G_{k}\left(i-j\right),\\ r_{k}=\sum_{i=1}^{L}\sum_{i=1}^{L}G_{k}\left(i-j\right)\left(\frac{\left(i-\mu_{i}\right)\left(j-\mu_{j}\right)}{\sqrt{\sigma_{i}^{2}\sigma_{j}^{2}}}\right). \end{array}$$

where

(8) $$\begin{array}{c} \mu_{i}=\sum_{j=1}^{L}\sum_{i=1}^{L}iG_{k}\left(i,j\right),\\ \mu_{j}=\sum_{j=1}^{L}\sum_{i=1}^{L}jG_{k}\left(i,j\right),\\ \sigma_{i}^{2}=\sum_{j=1}^{L}\sum_{i=1}^{L}{\left(i-\mu_{i}\right)}^{2}G_{k}\left(i,j\right),\\ \sigma_{j}^{2}=\sum_{j=1}^{L}\sum_{i=1}^{L}{\left(j-\mu_{j}\right)}^{2}G_{k}\left(i,j\right). \end{array}$$

Let the 4 × 1 vector *ν*_*k*_=[*c*_*k*_, *r*_*k*_, *e*_*k*_, *h*_*k*_]^*T*^ denote the feature vector for each channel; hence, the feature vector of each epoch considering all channels with 60 features is obtained as follows:

(9) $$\begin{array}{c} f_{60\times 1}={\left[\nu_{1}^{T},\ldots ,\nu_{15}^{T}\right]}^{T}. \end{array}$$

#### 3.2.3. Feature Selection

Selecting the best features among all obtained features plays a key role in the signal and image processing tasks [30, 38, 39]. In the previous part, we presented each EEG epoch with 60 features, but all computed features are not meaningful. Hence, significant features should be selected from the vector **f**. In this paper, we adopt the MRMR method [40]. Its goal is to find the set of features such that selected features are mutually and maximally dissimilar which is achieved by minimizing the redundancy and maximization of the relevance of the selected features to the actual classes. MRMR considers the pairwise mutual information of features and mutual information of a feature and actual classes to quantify the redundancy and relevance.

Let *r*_*h*_ and *e*_*h*_ denote the relevance of **h** with respect to a response **y** and the redundancy of **h**, respectively, which are defined as follows:

(10) $$\begin{array}{c} r_{h}=\frac{1}{\left|h\right|}\sum_{x\in h}I\left(x,y\right),\\ e_{h}=\frac{1}{{\left|h\right|}^{2}}\sum_{x,z\in h}I\left(x,z\right), \end{array}$$

where |**h**| is the cardinality of set **h** and *I*(*A*, *B*) is the mutual information of two sets *A* and *B* which is computed as follows:

(11) $$\begin{array}{c} I\left(A,B\right)=\sum_{i,j}P\left(A=a_{i},B=b_{j}\right)\log\frac{P\left(A=a_{i},B=b_{j}\right)}{P\left(A=a_{i}\right)P\left(B=b_{j}\right)}. \end{array}$$

The selected feature set **h** should maximize the *r*_*h*_ and minimize the *e*_*h*_. There are 2^|**f**|^combinations and finding the optimal set **h** requires them all. But, MRMR employs the forward addition scheme by using the mutual information quotient (MIQ) value to rank the features. MIQ value is defined as

(12) $$\begin{array}{c} q\left(f\right)=\frac{r_{f}}{e_{f}}, \end{array}$$

where *r*_*f*_ and *e*_*f*_ denote the relevance and redundancy of feature *f*, respectively, and defined as

(13) $$\begin{array}{c} r_{f}=I\left(f,y\right),\\ e_{f}=\frac{1}{\left|h\right|}\sum_{z\in h}I\left(f,z\right). \end{array}$$

The steps by which MRMR selects the features in the steps are as follows.

(1) Initialize the set of selected features as **h**={}.
(2) Select the feature with the largest relevance, *h*_1_=argmax_|**f**|_*r*_*f*_ and update **h** as **h**={*h*_1_}.
(3) Find the features with nonzero relevance and zero redundancy in the complement of **h**, i.e., **h**^*c*^.
  If **h**^*c*^ does not include a feature with nonzero relevance and zero redundancy, go to step 5.
  Otherwise, select the feature with the largest relevance, *h*=argmax_|**h**^*c*^|,*r*_*h*_=0_*r*_*f*_ and update **h** as **h**={**h**, *h*}
(4) Step 3 is repeated until the redundancy is greater than zero for all features in **h**^*c*^.
(5) Select the feature that has the largest MIQ value with nonzero relevance and nonzero redundancy in **h**^*c*^ and update **h** as **h**={**h**, *h*}
  (14) $$\begin{array}{c} h=\underset{h^{c}}{\arg\max}q_{h}=\underset{h^{c}}{\arg\max}\frac{I\left(h,y\right)}{\left(1/\left|h\right|\right)\sum_{z\in h}I\left(x,z\right)}. \end{array}$$
(6) Repeat step 5 until the relevance is zero for all features in **h**^*c*^.
(7) Add the features with zero relevance to **h** in random order.

### 3.3. Classification

The nonlinear and commonly used KNN classifier is considered in this paper to classify the features obtained from the feature selection step. KNN classifies the samples based on the distance between the unknown features and the features of training samples. It considers the labels of *K* as the most similar neighbors to predict the class of the training samples and considers the label of the class with the greatest number of samples among them [41–44]. In this study, we consider several distance measures to compute the similarity between the test and training samples.

Consider two feature vectors with *N* features as **v**={*v*_1_,…,*v*_*N*_}^*T*^and **w**={*w*_1_,…,*w*_*N*_}^*T*^. The different distance metrics are calculated as follows:

(i) Euclidean distance:
  (15) $$\begin{array}{c} d_{E}=\sqrt{{\left(v-w\right)}^{T}\left(v-w\right)}. \end{array}$$
(ii) Standardized Euclidean distance:
  (16) $$\begin{array}{c} d_{\text{SE}}=\sqrt{{\left(v-w\right)}^{T}V^{-1}\left(v-w\right)}, \end{array}$$
where *V* denotes the diagonal *N* × *N* matrix. The ith diagonal element of *V* is *S*^2^(*i*), where *S* is a vector of scaling factors for each dimension.
(iii) Minkowski distance:
  (17) $$\begin{array}{c} d_{mi}=\sqrt[{p}]{\sum_{i=1}^{N}{\left|v_{i}-w_{i}\right|}^{p}}. \end{array}$$
(iv) Chebyshev distance:
  (18) $$\begin{array}{c} d_{\text{ch}}=\underset{i}{\max}\left\{\left|v_{i}-w_{j}\right|\right\}. \end{array}$$
(v) City block distance:
  (19) $$\begin{array}{c} d_{\text{cb}}=\sum_{i=1}^{N}\left|v_{i}-w_{i}\right|. \end{array}$$
(vi) Cosine distance:
  (20) $$\begin{array}{c} d_{\text{cs}}=1-\frac{v^{T}w}{\sqrt{\left(v^{T}v\right)\left(\left(w^{T}w\right)\right)}}. \end{array}$$
(vii) Correlation distance:
  (21) $$\begin{array}{c} d_{\text{cr}}=1-\frac{{\left(v-\bar{v}\right)}^{T}\left(w-\bar{w}\right)}{\sqrt{{\left(v-\bar{v}\right)}^{T}\left(v-\bar{v}\right)}\sqrt{{\left(w-\bar{w}\right)}^{T}\left(w-\bar{w}\right)}}, \end{array}$$
where $\bar{v}$ and $\bar{w}$ are the mean of vectors **v** and **w**, which are computed as follows:
  (22) $$\begin{array}{c} \bar{v}=\frac{1}{N}\sum_{i=1}^{N}v_{i},\\ \bar{w}=\frac{1}{N}\sum_{i=1}^{N}w_{i}. \end{array}$$
(viii) Mahalanobis distance:
  (23) $$\begin{array}{c} d_{\text{ma}}=\sqrt{{\left(v-w\right)}^{T}C^{-1}\left(v-w\right)}, \end{array}$$
where **C** denotes covariance matrix.

It should be noted that, for *p*=1, *p*=2, and *p*=*∞*, Minkowski and the city block distances are the same, Euclidean distance, and Chebyshev distances, respectively.

## 4. Results

Here, we provide the obtained results to demonstrate the robustness of the proposed DoA classification, where a 10-fold cross-validation method is used to obtain the accuracy. In this way, the available data is randomly partitioned into 10 nonoverlapping parts with an equal number of samples, and training and testing procedure is repeated 10 times. At each time, nine parts are considered as training samples and one part is used for testing. Also, training and test are performed for each subject separately, and the results are reported for each subject.

In order to increase the number of training samples and enhancing the generality of the trained classifier, the data augmentation scheme is presented in [45]. This method increases the number of training samples by adding zero-mean Gaussian noise with standard deviation *σ* to them. It should be noted that data augmentation is only performed on training samples, and test samples are those selected from original samples. The classification accuracy is evaluated for several augmented multiples and noise variances.

### 4.1. Classification Accuracy

The classification accuracy of the proposed DoA classification is presented in Table 3 considering the features extracted from each channel of recorded EEG signals as well as considering whole features extracted from all channels. It is observed that the selection of the channel has considerable effect accuracy. These results are obtained considering augmented multiple and noise variance equal to 35 and 0.1, respectively. It should be noted that the performance of the proposed method is presented for different values of the augmented multiple and noise variances in the following subsections. Also, the number of gray levels is set to 16, and Mahalanobis distance is considered for measuring the distance between training and test samples.

It is observed that channel T7 provides the highest average accuracy which is equal to 75.54%. Also, subjects 4 and 6 have the highest accuracy as 67.93% and 82.41%, respectively. On the other side, channel Fz yields the lowest average accuracy at 65.63%, where subjects 4 and 2 have the lowest and highest accuracy equal to 52.29% and 77.98%, respectively.

According to reported results, considering whole extracted features from all channels enhances the classification accuracy considerably. In this case, the lowest and highest accuracy results belong to subjects 3 and 5 with 93.34% and 96.92%, respectively, and an average result of 95.32% is obtained. These results indicate the efficiency of the proposed method for the classification of EEG signals in order to determine DoA.

Table 4, in the revised version, compares the performances of several TFMs and classifiers. We considered the PWVD, WVD, and STFT as well as KNN, SVM, random forest, and decision tree classifiers. It is observed that the pair (SPWVD, KNN) outperforms the other pairs of TFMs and classifiers. For all TFMs, KNN provides the best accuracy, and then SVM yields good performance. Among TFMs, SPWVD and WVD have the highest and lowest accuracy, respectively.

### 4.2. Confusion Matrix

Table 5 presents the confusion matrix of the proposed method for the classification of DoA for different subjects. It is observed that the proposed method provides efficient accuracy for all subjects in the presence of biased data. It is noticeable that the proposed method does not classify the deep hypnotic as sedation and awake epoch and vice versa, which indicates the efficiency of the proposed method. The misclassifications of epochs from classes deep hypnotic and sedation and awake are classified as class surgical anesthesia. Also, most misclassifications of epochs from surgical anesthesia are classified as sedation and awake. The sensitivity of different classes is also provided in Table 4 which indicates the classification accuracy of each class in different subjects.

### 4.3. The Effect of the Number of Gray Levels

The effect of the number of gray levels in computing GLCM on the performance of the proposed DoA classification is presented in Table 6 in which the classification accuracy is obtained considering all channels. It is observed that, for all subjects, accuracy increases considerably as the number of gray levels increases from four to 16 while increasing the number of gray levels from 16 to 64 reduces the accuracy. Hence, 16 gray levels are considered in order to extract texture-based features from time-frequency images obtained from SPWVD.

### 4.4. Accuracy of Distance Measures

The accuracy of the proposed method considering different distance measures considered in the KNN classifier is given in Table 7. As mentioned earlier, the Mahalanobis distance provides the highest accuracy of 95.32%, and after that, the Chebyshev distance reaches the accuracy of 93.26%. Also, the standardized Euclidean distance has the lowest accuracy of 90.73%.

### 4.5. The Effect of Augmentation

The effect of the augmentation multiple and noise variances in data augmentation on the performance of the proposed DoA classification is shown in Figure 8, where the average accuracy of all subjects is reported. As observed from Figure 8(a), increasing the augmentation multiple from 1 to 35 increases the accuracy, but after that, accuracy reduces. Hence, the augmentation multiple is set to 35 in all results reported previously in this section. When the greater number of augmented data increases, it is possible that there is outlier data which reduces the accuracy. Also, it is seen from Figure 8(b) that increasing the noise variance from 0.1 to 0.1 increases the accuracy, but after that, accuracy reduces; therefore, we choose the variance of 0.1.

## 5. Conclusion

In this paper, we presented a noninvasive method for monitor the DoA based on time-frequency analysis of EEG signals recorded in 15 channels considering the electrode placement in 10/20 standard. EEG signals were recorded from six subjects and were partitioned into epoch with the length of 30 seconds, where consequent epochs have 50% overlap with each other. The TFM of each channel was calculated using SPWVD. Obtained TFM showed that frequencies higher than 8 Hz have near-zero amplitude, and we can remove them from TFM. Then, GLCM was employed to describe the gray content of each TFM. Contrast, correlation, energy, and homogeneity were calculated for each GLCM; hence, the feature vector of each epoch was constructed by 60 features. The redundant features were removed by the MRMR algorithm and KNN classified the remaining feature to determine the DoA. The results showed that the proposed method achieves the average accuracy of 95.32% with 16 gray levels and Mahalanobis distance and the minimum and maximum accuracy among subjects are 93.34% and 96.92%, respectively. The accuracy with high mean and low variation among subjects indicates the efficiency of the proposed method. We also analyzed the effect of the parameters of data augmentation, which indicates that augmentation multiple and noise variance equal to 35 and 0.1, respectively, achieve the highest accuracy.

Employing the methods based on deep learning and transfer learning can be considered as future works. Convolutional neural networks (CNNs) to classify the TFM are obtained from time-frequency analysis. From the viewpoint of time-series analysis, we can use long short-term memory (LSTM) networks to determine the DoA.

## Figures and Tables

**Figure 1:** The procedure of the presented method in this paper for DoA classification.

**Figure 2:** Signals of different channels in overdeep (D) class.

**Figure 3:** Signals of different channels in surgical anesthesia (A) class.

**Figure 4:** Signals of different channels in sedation and awake (S) class.

**Figure 5:** The SPWVD of different channels in overdeep (D) class.

**Figure 6:** The SPWVD of different channels in surgical anesthesia (A) class.

**Figure 7:** The SPWVDs of different channels in sedation and awake (S) class.

**Figure 8:** Accuracy of the proposed method for different values of (a) augmentation multiple and (b) noise variance.

**Table 1:** EEG recording duration for different patients.

Patient number	1	2	3	4	5	6
Duration (minutes)	90	140	140	52	175	105

**Table 2:** The number of epochs from each label for different patients.

Label	Patient					
	1	2	3	4	5	6
D	65	125	101	31	242	303
A	336	304	333	158	275	169
S	36	207	227	73	165	74
Total	437	636	661	262	682	546

**Table 3:** Classification accuracy of the proposed DoA classification.

Channel	Subject						Average	Min	Max
	1	2	3	4	5	6			
1 (Fp1)	77.80	65.72	68.68	55.72	74.48	83.51	70.98	55.72	83.51
2 (Fp2)	66.36	73.58	64.44	70.99	67.44	75.64	69.74	64.44	75.64
3 (F7)	65.21	74.37	64.75	61.83	77.41	74.35	69.65	61.83	77.41
4 (F3)	67.27	79.08	63.08	57.25	66.42	69.41	67.08	57.25	79.08
5 (Fz)	64.53	77.98	62.02	52.29	70.67	66.30	65.63	52.29	77.98
6 (F4)	69.56	63.36	73.97	50.76	74.34	82.41	69.07	50.76	82.41
7 (F8)	79.40	66.03	63.84	60.67	59.97	73.62	67.25	59.97	79.40
8 (T7)	73.22	79.24	69.74	67.93	79.03	84.06	75.54	67.93	84.06
9 (C3)	64.98	60.84	76.85	70.61	68.47	84.79	71.09	60.84	84.79
10 (Cz)	69.10	79.24	77.91	67.93	57.33	78.20	71.62	57.33	79.24
11 (C4)	67.73	71.06	68.38	53.81	76.39	81.86	69.87	53.81	81.86
12 (T8)	67.96	72.32	56.88	67.93	62.17	69.04	66.05	56.88	69.04
13 (P3)	73.68	64.62	72.31	54.19	62.31	78.75	67.64	54.19	78.75
14 (Pz)	69.56	63.99	66.26	68.32	73.61	74.35	69.35	63.99	74.35
15 (P3)	77.34	76.25	75.34	51.52	67.88	81.68	71.67	51.25	81.68
All	94.5	94.65	93.34	95.8	96.92	96.7	95.32	93.34	96.92

**Table 4:** Performance comparison between different TFMs and classifiers.

TFM	Classifier			
	KNN	SVM	Random forest	Decision tree
SPWVD	95.32	94.54	93.49	93.86
PWVD	94.01	93.46	92.34	92.80
WVD	93.24	92.52	91.35	92.00
STFT	93.70	93.11	91.59	92.18

**Table 5:** Confusion matrix of the proposed DoA classification.

		Predicted class			Sensitivity (%)
		D	A	S	
Actual class for subject 1	D	60	5	0	92.31
	A	4	320	12	95.24
	S	0	3	33	91.67

Actual class for subject 2	D	119	6	0	95.2
	A	7	285	12	93.75
	S	0	9	198	95.65

Actual class for subject 3	D	94	7	0	93.07
	A	12	311	10	93.39
	S	0	15	212	93.39

Actual class for subject 4	D	30	1	0	96.77
	A	2	151	5	95.57
	S	0	3	70	95.89

Actual class for subject 5	D	235	7	0	97.11
	A	4	264	7	96
	S	0	3	162	98.18

Actual class for subject 6	D	293	10	0	96.69
	A	2	163	4	96.45
	S	0	2	72	97.29

**Table 6:** The effect of the number of gray levels of GLCM.

Number of gray levels	Subject						Average	Min	Max
	1	2	3	4	5	6			
4	87.87	86.16	87.74	85.49	90.89	89.56	87.95	85.49	90.89
8	90.85	92.45	91.22	91.22	93.11	91.75	91.77	90.85	92.45
16	94.5	94.65	93.34	95.8	96.92	96.7	95.32	93.34	96.92
32	93.13	94.03	92.58	94.27	95.61	95.78	94.23	92.58	95.78
64	92.22	93.55	92.13	92.36	93.41	94.87	93.09	92.13	94.87

**Table 7:** Accuracy of different distance measures.

Distance measure	Subject						Average	Min	Max
	1	2	3	4	5	6			
Euclidean	93.59	91.98	93.34	89.69	94.87	92.67	92.69	89.69	94.87
Standardized Euclidean	89.02	91.04	91.38	92.37	89.69	90.84	90.73	89.02	92.37
Mahalanobis	94.50	94.65	93.34	95.80	96.92	96.70	95.32	93.34	96.92
City block	88.79	93.55	91.98	92.37	95.31	93.96	92.66	88.79	95.31
Minkowski	90.85	92.77	93.65	90.84	90.91	93.41	92.07	90.85	93.65
Chebyshev	94.28	92.92	90.47	90.46	94.72	96.70	93.26	90.46	96.7
Cosine	90.62	93.40	89.11	93.51	90.32	93.04	91.67	89.11	93.51
Correlation	92.45	93.87	89.86	91.60	96.92	93.96	93.11	89.86	96.92
Average	91.76	93.02	91.64	92.08	93.71	93.91			
Min	89.02	91.04	89.11	89.69	89.69	90.84			
Max	94.50	94.65	93.34	95.80	96.92	96.7			

## Data Availability

Data used to support the study are available from the corresponding author upon reasonable request.
